This article has been retracted.

# Development and Optimization of a Prognostic Model Associated with Stemness Genes in Hepatocellular Carcinoma

**DOI:** 10.1155/2022/9168441

**Published:** 2022-10-05

**Authors:** Kefen Zhang, Kaisheng Xie, Xin Huo, Lianlian Liu, Jilin Liu, Chao Zhang, Jun Wang

**Affiliations:** ^1^Guangxi University of Science and Technology, Liuzhou 545006, China; ^2^Department of Pathology, Second Affiliated Hospital of Guangxi University of Science and Technology, Liuzhou 545006, China; ^3^Department of Oncology, Liuzhou People's Hospital Affiliated to Guangxi Medical University, Liuzhou 545006, China; ^4^College of Information Science and Engineering, Shandong Agricultural University, Tai'an 271000, China

## Abstract

Hepatocellular carcinoma (HCC) is one of the most lethal cancers worldwide, which is associated with a variety of risk factors. Cancer stem cells are self-renewal cells, which can promote the occurrence and metastasis of tumors and enhance the drug resistance of tumor treatment. This study aimed to develop a stemness score model to assess the prognosis of hepatocellular carcinoma (HCC) patients for the optimization of treatment. The single-cell sequencing data GSE149614 was downloaded from the GEO database. Then, we compared the gene expression of hepatic stem cells and other hepatocytes in tumor samples to screen differentially expressed genes related to stemness. R package “clusterProfiler” was used to explore the potential function of stemness-related genes. We then constructed a prognostic model using LASSO regression analysis based on the TCGA and GSE14520 cohorts. The associations of stemness score with clinical features, drug sensitivity, gene mutation, and tumor immune microenvironment were further explored. R package “rms” was used to construct the nomogram model. A total of 18 stemness-related genes were enrolled to construct the prognosis model. Kaplan-Meier analysis proved the good performance of the stemness score model at predicting overall survival (OS) of HCC patients. The stemness score was closely associated with clinical features, drug sensitivity, and tumor immune microenvironment of HCC. The infiltration level of CD8^+^ T cells was lower, and tumor-associated macrophages were higher in patients with high-stemness score, indicating an immunosuppressive microenvironment. Our study established an 18 stemness-related gene model that reliably predicts OS in HCC. The findings may help clarify the biological characteristics and progression of HCC and help the future diagnosis and therapy of HCC.

## 1. Introduction

Tumor heterogeneity is one of the main characteristics of HCC, which makes the progress of treatment slow [1, 2]. At present, there is still a lack of biomarkers and effective prognostic models for diagnosis, prognosis, and prediction of therapeutic efficacy of HCC. This further weakens the possibility of developing personalized treatment. Single-cell genomics is a powerful strategy to depict the complex molecular landscape of cancer. Recent studies on the relationship between HCC cells and stem cell markers showed that the expression of EPCAM can effectively distinguish between stemness HCC cells and nonstemness HCC cells [3].

Cancer stem cells (CSCs) are self-renewal cells, which can promote the occurrence and metastasis of tumors and enhance the drug resistance of tumor treatment [4]. Transcriptome-based studies in multiple tumors have revealed a significant link between tumor stemness and patient prognosis and tumor immune microenvironment [5–7]. Recent studies have confirmed the effect of tumor stemness on immune cells in tumor microenvironment, namely, tumor-associated macrophages (TAMs), myeloid-derived suppressor cell (MDSC), and CD8^+^ T cells. In turn, these immune cells also play an important role in maintaining tumor stemness, creating a malignant environment [8]. However, there are few studies on tumor stemness in HCC, especially the relationship between tumor stemness and immune microenvironment. In recent years, the tumor stemness has attracted much attention. The main characteristics of tumor stemness are the strong self-renewal ability and increased tumor heterogeneity [3–4]. Many studies have shown that tumor stemness plays an important role in tumor metastasis, differentiation, and drug resistance [9, 10]. For example, USP22 was reported to promote the stemness of HCC cells by HIF1a pathways [11]. In addition, RALYL could increase HCC stemness via sustaining the mRNA stability of TGF-beta2 [12]. HDAC11, AMD1, and SENP1 were also proved to promote the stemness of HCC cells [13–15]. However, the proven stemness-related genes are far from enough in HCC. Thus, it is necessary and urgent to screen stemness genes and construct the stemness-related prognosis model in HCC.

In our study, we downloaded the single-cell sequencing data GSE149614 to screen stemness genes by comparing the gene expression difference of hepatic stem cells and other hepatocytes. R-package “clusterProfiler” was used to explore the potential function of stemness-related genes. We then constructed a prognostic model using LASSO regression analysis based on the TCGA and GSE14520 cohorts. The associations of stemness score with clinical features, drug sensitivity, gene mutation, and tumor immune microenvironment were further explored. R package “rms” was used to construct nomogram model. Our study defined stemness-related genes and constructed stemness-related prognostic model, which may support new ideas for screening therapeutic targets to inhibit stem characteristics and the development of HCC.

## 2. Materials and Methods

### 2.1. Data Collection

The single-cell sequencing data GSE149614 and RNA array data GSE14520 were downloaded from GEO database (https://www.ncbi.nlm.nih.gov/gds). The RNAseq data and clinical information of TCGA were obtained from the UCSC Xena database (https://xenabrowser.net/datapages/). In GSE149614, we extracted the data of primary HCC and adjacent tissues for follow-up analysis, including 18 samples (10 cancer tissues, 8 adjacent tissues) and 63101 cells. In GSE14520, after removing the samples with nontumor and incomplete prognostic data, a total of 225 samples were enrolled for subsequent analysis. In TCGA, We selected 362 tumor samples with survival data for follow-up analysis.

### 2.2. Identification of Stemness-Related Genes

Based on the single-cell transcriptome sequencing data of GSE149614, the expression data were quality controlled, standardized, and clustered using the R package “Seurat” (v4.0.5). According to the expression of EPCAM (epithelial cell adhesion molecule) gene, we identified the liver stem cell population and hepatocytes according to the cell annotation information provided by the references [16]. Then, we compared the gene expression of hepatic stem cells and other hepatocytes in tumor samples to screen differential expressed genes related to stemness. Further, we used R-package “clusterProfiler” (v4.0.5) to perform the functional enrichment of stemness-related genes.

### 2.3. Construction of Prognosis Model of HCC

Based on stemness-related genes, LASSO (least absolute shrinkage and selection operator) regression analysis was conducted. The stemness-related genes related to prognosis were screened, and the prognostic risk assessment model was constructed. In order to improve the accuracy of the model, we first filter out the feature factors with high correlation, and the threshold is 0.8. The model construction is based on the R package “glmnet” (v4.1-2), and 10-fold cross-validation is selected. We finally constructed a prognostic risk prediction model containing 18 stemness-related genes. The model is as follows:

Stemness Score = AKR1B10∗0.02688 + AKR1C3∗0.0214 + BSG∗0.05855 + CD74∗(−0.07195) + CLDN6∗0.17068 + CYP3A5∗(−0.01822) + GLB1∗0.005275 + HSP90AA1∗0.12853 + HSPA6∗0.002546 + KRT19∗(−0.02418) + MIF∗(−0.02593) + NQO1∗0.015396 + NUPR1∗0.056 + PDCD6IP∗0.01709 + PHLDA2∗0.02894 + PON1∗(−0.06318) + RANBP1∗0.41467 + SLC2A2∗(−0.02551).

Furthermore, a nomogram was constructed using the R package “rms.”

### 2.4. Statistical Analysis

Based on the expression profile data of TCGA-LIHC, the immunotherapy efficacy prediction software TIDE (http://tide.dfci.harvard.edu/) was used to predict the efficacy score of immunotherapy. The differences of efficacy score between the high- and low-stemness score groups were compared. We also compare the expression of immune checkpoints (PD1, PD-L1, CTLA4) between the high- and low-stemness score groups. The R package “CIBERSROT” was used to calculate the proportion of 22 immune cells. The R package “ESTIMATE” was used to evaluate the stromal, immune, and tumor purity scores using the TCGA-LIHC data. We also calculated the score of HALLMARK pathways using the R package “GSVA.” The HALLMARK pathways were downloaded from the MSigDB database (http://www.gsea-msigdb.org/gsea/msigdb/collections.jsp).

Based on the expression data of TCGA-LIHC, the R package “pRRophetic” (v0.5) was used to predict the sensitivity of chemotherapy and targeted therapeutic drugs (half maximal inhibitory concentration: IC50) for HCC patients. The differences of IC50 between the high- and low-stemness score groups were compared. The independent Student's t-test for continuous data and the *Х^2^* test for categorical data were utilized for pairwise comparisons between groups. The Mann-Whitney *U* test was used to compare categorical variables and nonnormally distributed variables between two groups. The Kruskal-Wallis test was used to compare multiple groups. Correlations between normally distributedvariables were assessed with Pearson's correlation test, while correlationsbetween nonnormally distributed variables were assessed with Spearman's correlation test. The statistical analyses in this study were performed by using R 4.1.0 software. A two-tailed *P* value <0.05 was considered statistically significant.

## 3. Results

### 3.1. Identification of Stemness-Related Genes

First, we downloaded the single-cell sequencing data GSE149614 from the GEO database.  Figure 1 displays the expression and distribution of genes, cells and mitochondria genes. All the cells were classified into 53 types (Figure 2(a)), in which there were significant differences in the cell community structure between tumor tissues and noncancer tissues. More types of cells and dispersion were observed in tumor tissues (Figure 2(b)). We use the cell annotation information provided by references.  Figure 2(c) displays the results of cell annotation. We found that the noncancerous tissue cells are mainly T/NK cells, myeloid cells, and endothelial cells. Epithelial cell adhesion molecule (EPCAM) is a marker of human liver stem cells (HSC) and progenitor cells, which does not exist in mature hepatocytes. However, EPCAM is also expressed in tumors and damaged liver. In the single-cell transcriptome sequencing data of liver cancer, EPCAM is mainly expressed in tumor cells and concentrated in cluster10 (Figures 2(b) and 2(d)).

Liver cells in tumor tissues are mainly annotated as 9 categories, namely, cluster2, cluster4, cluster7, cluster10, cluster14, cluster17, cluster20, cluster34, and cluster37. We further screened 145 differential expressed genes, which were considered as stemness-related genes, between cluster10 and other 8 clusters (Figure 3). Heatmap presents differential expressed genes. HSC represents liver stem cells, and HPC represents other hepatocytes.

### 3.2. Enrichment Analysis of Stemness-Related Genes

We also explored the function of 145 stemness-related genes. Results indicated that stemness-related genes were mainly enriched in fatty acid metabolic process and alcohol metabolic process in biological process (BP) (Figure 4(a)), blood microparticle and collagen-containing extracellular matrix in cellular components (CC) (Figure 4(b)), carboxylic acid binding and oxidoreductase activity, acting on CH-OH group of donors in molecular function (MF) (Figure 4(c)), and metabolism of xenobiotics by cytochrome P450 and chemical carcinogenesis-reactive oxygen species in KEGG (Figure 4(d)).

### 3.3. Construction of Prognosis Prediction Model of HCC

To construct a prognosis prediction model of HCC based on 145 stemness-related genes, we conducted lasso regression analysis using TCGA-LIHC as training cohort and GSE14520 as validation cohort. Finally, 18 stemness-related genes were enrolled to construct the prognosis model. Based on the prognosis model, we calculated the stemness score of each sample and found that patients with high-stemness score have worse survival status in TCGA-LIHC (Figure 5(a)) and GSE14520 cohorts (Figure 5(b)).

### 3.4. The Association of Stemness Score with Clinical Characters, Gene Mutation, and Drug Resistance of HCC Patients

We further explored the association of stemness scores with clinical characters of HCC patients using the TCHA-LIHC cohort (Figure 6(a)). We found that stemness score was significantly correlated with the survival status of patients, and stemness score was higher in the dead patient group (Figure 6(b)). There were no correlation of stemness score with age, gender, and race (Figures 6(c)–6(e)). Stemness score was significantly higher in stage III patients than in stage I patients (Figure 6(f)). In addition, we found that there was a significant correlation between stemness score and tumor histological grade. The higher the grade, the higher the stemness score (Figure 6(g)).  Figure 6(h) shows that stemness score in obese people with BMI greater than 30 is significantly lower than that in normal people with BMI ≤25.

We then analyzed the correlation between stemness score and tumor mutation load (Figure 7(a)) and found that stemness score was higher in group with high mutation load (Figure 7(b)). In addition, there was a significant correlation between TP53 mutation status and stemness score in HCC. Stemness score in the mutant group was significantly higher than that in the wild-type group (Figure 7(c)). There was no association of stemness score with mutation of CTNNB1, ARID1A, ARID2, PCLO, AXIN1, and APOB (Figures 7(d) and 7(e)).

Besides, we compared the gene mutation frequency in the high- and low-stemness score group. Results indicated that the mutation frequency of TP53 was the highest in the high-stemness score group, while the mutation frequency of CTNNB1 was the highest in the low-stemness score group (Figures 8(a) and 8(b)). The oncoplot displays the gene mutation frequency in the high- and low-stemness score group.

To explore the relationship between stemness score and tumor drug resistance, we predicted the IC50 of anti-cancer drugs using the R package “pRRophetic” based on the TCGA-LIHC cohort. We found that there were significant differences in the sensitivity of patients to cisplatin, gemcitabine, and gefitinib, in which the IC50 was lower in the high-stemness score group (Figures 9(a), 9(c), and 9(d)). These results indicated that patients with high-stemness score may be more sensitive to cisplatin, gemcitabine, and gefitinib treatment. In addition, the IC50 value of erlotinib was higher in the high-stemness score group, suggesting that HCC patients with high-stemness score may be more resistant to erlotinib treatment (Figure 9(b)).

### 3.5. The Association of Stemness Score with Tumor Immune Microenvironment

Since there was no publicly available immunotherapy dataset of HCC, we used the TIDE database to predict the efficacy score of immunotherapy based on the TCGA-LIHC cohort. We found that the TIDE score was higher in the high-stemness score group, suggesting a poor therapeutic effect of immune checkpoint inhibitors (Figure 10(a)). In addition, CTLA4 and PDCD1 were highly expressed in the high-stemness score group (Figure 10(b)). There was no significant difference of CD274 (Figure 10(c)).

We further explored the association of stemness score with immune cell infiltration. The infiltration level of CD8^+^ T cells and monocytes in the high-stemness score group was significantly lower than that in the low-stemness score group, while the infiltration level of macrophage M0, memory B cells, and eosinophils in the high-stemness score group were significantly higher than that in the low-stemness score group (Figure 11(a)). Further, the stemness score was positively correlated with macrophage M0 and negatively correlated with CD8^+^ T cells (Figure 11(b)). In addition, we observed a slight negative correlation of stemness score with stromal score (Figure 11(c)) and no significant correlation of stemness score with tumor purity, immune score, and ESTIMATE score (Figures 11(d)–11(f)).

### 3.6. The Correlation between Stemness Score and HALLMARK Pathways

Then, we explored the correlation between stemness score and HALLMARK pathways. We found that the pathways related to cell replication (MITOTIC_SPINDLE, MYC_TARGETS_V1, G2M_CHECKPOINT, E2F_TARGETS, DNA_REPAIR, and MYC_TARGETS_V2) were more active in the high-stemness score group, and the pathways related to material/energy metabolism (CHOLESTEROL_HOMEOSTASIS, COAGULATION, PEROXISOME, FATTY_ACID_METABOLISM, XENOBIOTIC_METABOLISM, BILE_ACID_METABOLISM, ADIPOGENESIS, and OXIDATIVE_PHOSPHORYLATION) were more active in low-stemness score group (Figure 12). These phenomena suggested that the tumor tissues of the two groups of samples are in significant different status, indicating that our model is of great significance in the risk stratification of tumor prognosis. Heatmap displays the GSVA score of HALLMARK pathways in TCGA cohort.

### 3.7. Construction of Nomogram Model of HCC

Finally, we constructed a nomogram to quantify patient risk based on stemness score and clinical characteristics of HCC patients. ROC curves were used to estimate the predictive ability of the model for prognosis. The nomogram based on TCGA-LIHC showed that the stemness score was a risk factor for the prognosis of HCC. The area under curve (AUC) values of 1-, 3-, and 5-year survival were 0.827, 0.74, and 0.724, respectively (Figures 13(a) and 13(b)). In GSE14520, we also proved that the stemness score was a risk factor for the prognosis of HCC. The area under curve (AUC) values of 1-, 3-, and 5-year survival in GSE14520 were 0.682, 0.648, and 0.615, respectively (Figures 13(c) and 13(d)).

## 4. Discussion

Tumor heterogeneity is one of the main characteristics of HCC, which makes the progress of treatment slow [1, 2]. At present, there is still a lack of biomarkers and effective prognostic models for diagnosis, prognosis, and prediction of therapeutic efficacy of HCC. This further weakens the possibility of developing personalized treatment.

In our work, we firstly downloaded the single-cell sequencing data GSE149614 from GEO database. We found that EPCAM is mainly expressed in tumor cells and concentrated in cluster10. We further screened 145 differential expressed genes, which were considered as stemness-related genes, between stemness HCC cells and nonstemness HCC cells. Enrichment analysis indicated that stemness-related genes were mainly enriched in fatty acid metabolic process and alcohol metabolic process in BP, blood microparticle, and collagen-containing extracellular matrix in CC, carboxylic acid binding and oxidoreductase activity, acting on CH-OH group of donors in MG, and metabolism of xenobiotics by cytochrome P450 and chemical carcinogenesis-reactive oxygen species in KEGG. We also conducted LASSO regression analysis using TCGA-LIHC as training cohort and GSE14520 as validation cohort to construct a prognosis prediction model in HCC. Patients with high-stemness score have worse survival status in the TCGA-LIHC and GSE14520 cohorts. We further explored the association of stemness score with clinical characters of HCC patients and found that stemness score was higher in the dead patient group. In addition, the higher the grade of HCC, the higher the stemness score. There was also a significant correlation between TP53 mutation status and stemness score in HCC.

We further explored the association of stemness score with immune cell infiltration. The infiltration level of CD8^+^ T cells and monocytes in the high-stemness score group was significantly lower than that in the low-stemness score group, while the infiltration level of macrophage M0, memory B cells, and eosinophils in the high-stemness score group was significantly higher than that in the low-stemness score group. These results suggested that patients with high-stemness score may have immunosuppressive tumor microenvironment.

Finally, we constructed a nomogram to quantify patient risk based on stemness score and clinical characteristics of HCC. The nomogram based on TCGA-LIHC showed that the stemness score was a risk factor for the prognosis of HCC. The area under curve (AUC) values of 1-, 3-, and 5-year survival were 0.827, 0.74, and 0.724, respectively. In GSE14520, we also proved that the stemness score was a risk factor for the prognosis of HCC. The area under curve (AUC) values of 1-, 3-, and 5-year survival in GSE14520 were 0.682, 0.648, and 0.615, respectively.

In conclusion, our study defined stemness-related genes and constructed stemness-related prognostic model, which may help clarify the biological characteristics and progression of HCC and help the future diagnosis and therapy of HCC. However, there are some limitations in our study such as insufficient experiments to explore the detailed function of stemness-related prognostic model. In the future, we need to conduct experiments to verify the influence of stemness-related prognostic mode on clarifying the biological characteristics and progression of HCC.

## Figures and Tables

**Figure 1:** The expression distribution of single cell transcriptome.

**Figure 2:** Cell clustering of GSE149614. (a) tSNE diagram shows the total clustering. (b) tSNE diagram shows the distribution of tumor cells and normal cells. (c) Cell annotation results. (d) The distribution of EPCAM.

**Figure 3:** Differentially expressed genes.

**Figure 4:** Enrichment analysis of stemness-related genes. (a) Top 20 results of GO enrichment analysis in BP terms. (b) Top 20 results of GO enrichment analysis in CC terms. (c) Top 20 results of GO enrichment analysis in MF terms. (d) Top 20 results of KEGG enrichment analysis.

**Figure 5:** The survival analysis of stemness gene model. Kaplan-Meier curves of stemness gene model in TCGA-LIHC cohort (a) and GSE14520 cohort (b).

**Figure 6:** Correlation analysis between stemness score and clinical characteristics. (a) Heatmap displays the correlation between stemness score and clinical characteristics. (b–h) The stemness score in indicated groups of various clinical characteristics.

**Figure 7:** Correlation analysis between stemness score and gene mutation. (a) Heatmap displays the correlation between stemness score and gene mutation. (b–i) The stemness score in indicated groups of various gene mutation status.

**Figure 8:** Oncoplot of gene mutation.

**Figure 9:** The correlation of stemness score with drug sensitivity. (a–d) The IC50 value of indicated drugs in the high- and low-stemness score group ∗∗ means *P* < 0.01,∗∗∗ means *P* < 0.001.

**Figure 10:** The association between stemness score and immunotherapy. (a–d) The TIDE score, CTLA4, CD274, and PDCD1 expressions in the high- and low-stemness score group.

**Figure 11:** The correlation of stemness score with immune cell infiltration. (a) The immune cell infiltration level in the high- and low-stemness score group. (b) The correlation of stemness score with immune cell infiltration level. The correlation between stemness score and stromal score (c), tumor purity (d), immune score (e), and ESTIMATE score (f) ‘ns' means *P* < 0.05, ∗ means *P* < 0.05, ∗∗ means *P* < 0.01, ∗∗∗ means *P* < 0.001, ∗∗∗∗ means *P* < 0.0001.

**Figure 12:** GSVA of stemness score.

**Figure 13:** Construction of nomogram model. (a) The nomogram in TCGA-LIHC cohort. (b) The ROC curves in TCGA-LIHC cohort. (c) The nomogram in GSE14520 cohort. (d) The ROC curves in GSE14520 cohort.

## Data Availability

The data sets analyzed during the current study are available from the corresponding author on reasonable request.
